# Altitudinal distribution and seasonal migration of asiatic black bear (*Ursus thibetanus*) in kaghan and Siran Valleys, Pakistan

**DOI:** 10.1016/j.heliyon.2023.e18052

**Published:** 2023-07-07

**Authors:** Zaib Ullah, Amir Said, Abdul Majid Khan, Asad Ullah, Shumaila Noreen, Sajid Mahmood

**Affiliations:** a School of Life and Environmental Sciences, Faulty of SEBE, Deakin University Waurn Ponds Campus, Victoria 3216, Australia; b Department of Zoology, Hazara University Sub-Campus Battagram, Khyber Pakhtunkhwa, Pakistan; c Institute of Zoology, University of the Punjab, Lahore 54590, Pakistan; d Department of Zoology, Hazara University Mansehra, Khyber Pakhtunkhwa, Pakistan; e Department of Zoology, University of Chakwal, Punjab, Pakistan

**Keywords:** altitudinal distribution, Seasonal migration, Sign survey, Transect, *Ursus thibetanus*

## Abstract

The Asiatic black bear (*Ursus thibetanus*) is considered one of the largest carnivores inhabiting different territories including coniferous and broad-leaved forests, extending from sea level to the elevation of 4300 m. The Kaghan and Siran Valleys in Pakistan's District Mansehra were the location of the current study. To evaluate the altitudinal distribution and seasonal movement of Asiatic black bears in the region, we used three approaches (sign distribution survey, questionnaire-based survey, and scat collecting). A total of 1858 bear signs were observed during the field survey, the highest number of signs was dig marks (1213) followed by plant uprooting. Dig marks (MER: 7.574) were observed repeatedly in each potential site of both valleys followed by plant uprooting (MER: 1.594). Similarly, the altitudinal distribution of black bears was determined through the frequency of signs concerning elevation (m). Elevation of the study area ranged from 1300 to 3500 m and the most abundant population was recorded at the elevation of 2501–3000 m followed by 2001–2500 m. About 52% of local communities encountered black bears during the summer season in the field followed by Spring (23%.8) and winter (15.3%). Manshi Reserver forest (24.5%) from Kaghan and Panjul Reserve forest (31.6) from Siran Valley are the potential summer migratory spots. Eleven scat samples were collected with a 0.103 encounter rate (ER). Most of the scats (about 70%) were observed within the maize crop field in the summer season at low elevation, while just 30% of the scat was observed in the winter season in the forest.

## 1 Introduction

Fossils records and ancient perception indicated the presence of sixteen bear species and presently eight bear species are testified globally viz; Brown bear (*Ursus arctos*), Giant Panda (*Ailuropoda melanoleuca*), American black bear (*Ursus americanus*), Sun bear (*Helarctos malayanus*), Sloth bear (*Melursus ursinus*), Polar bear (*Ursus maritimus*) and Asiatic black bear (*Ursus thibetanus*) [1]. Of these species, six species in Asia, one in South America, two in Europe, and three species were found in North America, while black and brown bears are present in the Azad Jammu and Kashmir and the Northern area of Pakistan [2].

The largest carnivore, the Asiatic black bear was first reported from Germany and France but later on, it moved to Taiwan, Vietnam, Laos, Korea, Indo-china, Japan, India, Iran, Afghanistan, and Pakistan [[1], [2], [3], [4], [5], [6]]. Mostly the bear is resident to the moist temperate forests of Siran, Kaghan, and Neelum Valley, of Gilgit-Baltistan and Khyber Pakhtunkhwa and Gilgit-Baltistan Pakistan, whereas in the Suleman range the local inhabitant species of bear known as “Baluchistan Black Bear”, is also present [1,7].

Forests and shrubby areas are the preferred places of bears and also they are found in burn areas, plan areas, meadows, and wetlands [8]. Season-wise they alter their territory in search of food [1]. The body weight of a bear reaches double its size before hibernation and also collects sufficient foodstuff to pass the harsh snowy season [9]. Season-wise movement of bears is mostly because of their breeding activity, reproduction, denning, and diet [10], and during this migration, the bear uses the skills like game trails, human trails, edges, shorelines, and rivers [11].

The current research focuses on the altitudinal variation and seasonal migration of black bears in search of food sources, due to their random movement toward villages or highly populated areas where they are facing severe threats from local communities like hunting, retaliatory killing, and poisoning to protect local crops. This article indicates the potential finding about black bear threats due to migration in the Kaghan and Siran valleys of district Mansehra which is considered one of the best ecological zones for the bear population in Pakistan.

## 2 Materials and methods

### 2.1 Study area

This study was conducted in a very important ecological zone (Siran and Kaghan Valleys) (34.234°–35.184°N and 72.817° to 74.134°E) of Pakistan. The study area is surrounded by neighboring districts like Kohistan, Battagram, Abbottabad, Azad Jammu, Kashmir, and some parts of northern areas. Very rich fauna and flora have been reported in the area and are mainly composed of moist temperate forests with abundant biodiversity. Area of the Kaghan (22,000 ha) and Siran Valley (13,744 ha) while the total areas of both valleys are 35,744 ha, including Reserves and Guzara Forests (Fig. 1) [4,6,12].

**Fig. 1:** Study area; Siran and Kaghan Valleys of District Mansehra.

## 3 Methods

Data were collected from both community and reserved forests in both valleys from 2019 to 2021 under the Sustainable Forests Management (SFM) project. Each sampling survey was planned fortnightly to collect black bear signs, scats, and perceptions of locals towards the bear population. We followed three main methods (black bear sign survey, questionnaire survey and scat collection) which were used by Refs. [3,4,6,12] for data collection about the black bear population and risk management.

### 3.1 Black bear sign survey

The line transects method was followed in potential sites for searching various bear signs. The transect size varies from 100 to 500 m long, whereas the width is normally 10–20 m. During this methodology, three well-trained researchers were involved in which two of them moved in the zigzag direction to search for bear signs and one person on the med line to record the data. A total of 33 line transects were drawn in the entire study area, and the encounter rate was calculated for each category of the sign. The encounter rate was calculated with the help of this formula (number of sign/transect length). Different categories of signs were observed i.e. pug marks, tree marks, bark off, plants uprooting, claw marks, stone replacing, bite marks, hair samples, dig marks, honey bees hive damages, scat samples, coarse wood damages, crop damages, place of livestock killing and place of temporary setting were recorded [4,6,13].

### 3.2 Sighting of the black bear by the local community

A questionnaire-based survey was conducted about sighting information from the local community. Each questionnaire is composed of multiple questions about black bear distribution and seasonal migration to the low altitude areas seasonally. A total of 100 questionnaires were filled from different villages of both valleys where mostly black bears were observed in the field during the summer season at very low elevations [6,12].

### 3.3 Scat collections

During the collection scat samples of the bear were randomly picked with the help of gloves and were stored in zip-lock plastic bags. A descriptive data sheet was used to record the date, time, and location of the sample. The collected samples were named and were kept at −20 C° for further use [3,13].

## 4 Results

### 4.1 Altitudinal distribution of black bear signs

During the field study of both valleys, thirteen various types of marks were identified. These marks were used to identify the black bear's behavior. Along with that 1858 bear signs were collected in which the high sign mark was dig mark (1213) followed by plants uprooting (186) and claw marks (134) were observed (Fig. 2).

**Fig. 2:** Various signs of black bears in both valleys.

The Mean Encounter Rate (MER) was calculated for each sign. Among all types of signs, dig marks (MER: 7.574) were observed frequently in each potential site of both valleys followed by plant uprooting (MER: 1.594) and claw marks (MER: 1.029) (Fig. 3). The encounter rate of bear signs indicated that bear populations are present in both valleys quite abundantly. Similarly, the altitudinal distribution of black bears was determined from the frequency of these signs concerning elevation (m) from sea level. Elevation of both valleys ranged approximately from 1300 to 3500 m and the most abundant population (based on a sign survey) of a black bear was recorded at the elevation of 2501–3000 m followed by 2001–2500 m. The altitudinal distribution also indicated that the black bear population is smaller at low (below 1500 m) and high elevation (above 3500 m). The study area is one of the important ecological zones and moist temperate forest, which is why most of the bear population prefer normal elevation (2000–3000 m) where the rate of precipitation and moist are high, so plants species and food sources are also very diverse (Fig. 4).

**Fig. 3:** Mean Encounter rate (MER) of bear signs.

**Fig. 4:** Altitudinal distribution of all bear signs (Mean encounter rate) from both valleys.

### 4.2 Seasonal migration of black bear

A questionnaire-based survey was conducted from the selected local community who has encountered a black bear in various seasons. According to the perception of locals, among the four seasons, encountering black bears mostly happened in the summer season when black bears have been observed at low elevations because of crop availability. The mean average response was calculated from the questionnaire survey in the study area. About 52% of the local community encountered black bears during the summer season in the field followed by Spring (23%.8) and winter (15.3%) (Fig. 5). Among all the sites, Manshi Reserver forest (24.5%), followed by Malakandireserve forest (22.5%), Kamal Bann Reserve forest (20.0%), and Bhageer Guzara forest (15.4%) were considered the most potential sites of black bear in Kaghan valley concerning summer migration. Similarly, Panjul reserve forest (31.6%), Una Reserve Forest (24.6%), and Manda Ghucha Guzara forest (13.9%) from Siran Valley are the summer migratory spots. The local community of the study area claimed that black bears attack their fields and cause greater economic loss in terms of crops and livestock (1501–2500 m) in the summer season. In the winter season, black bears move towards bushy areas and find a suitable den for hibernation (2501–3000 m) (Fig. 6).

**Fig. 5:** Response of the local community towards seasonal encountering with black bear.

**Fig. 6:** Seasonal variation of black bear is associated with altitudinal distribution in both valleys.

### 4.3 Scat samples

Food materials are the best source to identify the black bear. During this field visit, 11 fresh scat samples were collected with a 0.103 encounter rate (ER), in which five samples (ER: 0.046) were from Siran and six samples (ER: 0.06) were from Kaghan Valley. Most of the scats (about 70%) were observed within the maize crop field in the summer season at low elevations, while just 30% of the scat samples were observed in the winter season in the forest.

## 5 Discussion

Asiatic black bear altitudinal distribution and migration were investigated by various studies in different countries. In Pakistan [14], investigated the altitudinal distribution and diet composition of Asiatic black bears in the western Himalayas region (Kaghan Valley only). Local villagers (n = 180) were interviewed about diet composition and signs of black bears (n = 178) in different elevations. Respondents point out that Asiatic black bears are mostly present in the Malkandi, Kamal Bann, and Jaraid forests, and regularly visit the agricultural fields that are located near villages at the edge of the forest. Scat samples were investigated for diet identification and interactions play a vital role in causing the human-black bear conflict in the area. Similarly, (Bista and Aryal, 2013) investigated that most of the signs of black bears were observed at 2301–2700 m (>40%) and, 2701–3100 m (>25%) above the sea level in Nepal. According to the present study, altitudinal distribution and seasonal migration of Asiatic black bears were investigated through a sign survey, Questionnaire-based survey, and scat sample identification in Kaghan and Siran valleys, District Mansehra, Pakistan. As a result of the sign survey, thirteen different types of signs were observed, and the Mean Encounter rate was calculated for each type of sign. Among all types of signs, dig marks (MER: 7.574) were observed frequently in each potential site of both valleys followed by plant uprooting (MER: 1.594) and claw marks (MER: 1.029). Similarly, the altitudinal distribution of black bears was determined from the frequency of these signs concerning elevation (m) from sea level. The elevation of the study area ranged approximately from 1300 to 3500 m and the most abundant population of black bear were recorded at the elevation of 2501–3000 m followed by 2001–2500 m. The study area is one of the important ecological zones and moist temperate forests which is why most of the bear population prefers normal elevation (2000–3000 m).

Scat identification and distribution is considered one of the most commonly used techniques to investigate the feeding ecology and the seasonal migration of large carnivores [15]. Another study [14] reported that due shortage of natural food in the forest areas, which are not sufficient for the black bear's energy requirements; consequently, black bears go towards the agricultural fields for crop riding to fulfil their need. More than 60% of the respondents respond to the crop-raiding by Asiatic black bears in Kaghan Valley. Similarly, Crop raiding, which includes the consumption of potato, maize, plum, peach, prune, banana, date palm, and papaya by Asiatic black bears, has been reported in various in Taiwan [16], China [17], and in Iran [[18], [19], [20]]. In our study, we investigated that Asiatic black bears show seasonal migration to lower elevated areas in both valleys. According to the perception of locals, encountering black bears mostly happened in the summer season when black bears have been observed at low elevations because of crop availability. About 52% of the local community encountered black bears during the summer season in the field followed by spring (23%.8) and winter (15.3%). Among all the sites, Manshi Reserve Forest (24.5%), followed by Malakand reserve forest (22.5%), Kamal Bann reserve forest (20.0%), and Bhageer guzara forest (15.4%) were considered the most potential sites of black bear in Kaghan valley concerning summer migration. Similarly, the Panjul reserve forest (31.6%), Una Reserve Forest (24.6%), and Manda Ghucha guzara forest (13.9%) from Siran Valley are the summer migratory spots potentially.

## 6 Conclusion

Altitudinal variation and seasonal migration assessment of Asiatic black bears were conducted in Kaghan and Siran Valleys, Pakistan. Elevation of the study area ranged from 1300 to 3500 m and the most abundant population was recorded at the elevation of 2501–3000 m followed by 2001–2500 m. According to the perception of locals, the encounter rate of a black bear was mostly observed in the summer season at low elevations because of crop availability. Asiatic black bear migration in the study area is remarkable, due to a shortage of natural food, black bears migrate to lower evaluated areas for crop-raiding in the summer season where severe Human-black bear conflict occurred. A very high level of conservation efforts and supplemental foods are recommended for the protection of black bears in one of the important ecological zones of Pakistan.

## Availability of data and materials

Data from this article is available for any sort of publicity after publication.

## Consent for publication

The author is agreed and signed for publication.

## Authors contribution

ZU: Conceived and designed the experiments, Analyzed and interpreted the data and Wrote the paper.

AS and AU: Analyzed and interpreted the data and Performed the experiments.

AMK, SN and SM: Contributed reagents, materials, analysis tools or data, Conceived and designed the experiments, and supervised the proposed the study.

## Declaration of competing interest

The authors declare that they have no known competing financial interests or personal relationships that could have appeared to influence the work reported in this paper.
